RETRACTED

# The Therapeutic Roles of Cinnamaldehyde against Cardiovascular Diseases

**DOI:** 10.1155/2022/9177108

**Published:** 2022-10-08

**Authors:** Li Lu, Yuan Xiong, Juan Zhou, Guangji Wang, Bobin Mi, Guohui Liu

**Affiliations:** ^1^Department of Orthopaedics, Union Hospital, Tongji Medical College, Huazhong University of Science and Technology, Wuhan 430022, China; ^2^Department of Cardiology, Hubei Provincial Hospital of Traditional Chinese Medicine, Wuhan 430073, China; ^3^Department of Cardiology, The Central Hospital of Wuhan, Tongji Medical College, Huazhong University of Science and Technology, Wuhan 430014, China

## Abstract

Evidence from epidemiological studies has demonstrated that the incidence and mortality of cardiovascular diseases (CVDs) increase year by year, which pose a great threat on social economy and human health worldwide. Due to limited therapeutic benefits and associated adverse effects of current medications, there is an urgent need to uncover novel agents with favorable safety and efficacy. Cinnamaldehyde (CA) is a bioactive phytochemical isolated from the stem bark of Chinese herbal medicine Cinnamon and has been suggested to possess curative roles against the development of CVDs. This integrated review intends to summarize the physicochemical and pharmacokinetic features of CA and discuss the recent advances in underlying mechanisms and potential targets responsible for anti-CVD properties of CA. The CA-related cardiovascular protective mechanisms could be attributed to the inhibition of inflammation and oxidative stress, improvement of lipid and glucose metabolism, regulation of cell proliferation and apoptosis, suppression of cardiac fibrosis, and platelet aggregation and promotion of vasodilation and angiogenesis. Furthermore, CA is likely to inhibit CVD progression via affecting other possible processes including autophagy and ER stress regulation, gut microbiota and immune homeostasis, ion metabolism, ncRNA expression, and TRPA1 activation. Collectively, experiments reported previously highlight the therapeutic effects of CA and clinical trials are advocated to offer scientific basis for the compound future applied in clinical practice for CVD prophylaxis and treatment.

## 1. Introduction

In the past decade, cardiovascular diseases (CVDs) contributed the most to mortality and disability across the world, accounting for an estimated 18 million fatalities annually. According to the WHO statistics, more than 500 million people were suffering from CVDs in 2019, which is approximately double that in 2009 [1–3]. The number of CVDs patients has rapidly increased recently mostly because of the lack of physical exercise, consumption of high calorie diet, air pollution, and other factors [1, 4]. As numerous pathogenic events, such as inflammatory response and oxidative stress, as well as highly prevalent predisposing threats, such as diabetes and obesity, are associated with CVDs, the effects of currently available drugs on the prevention and treatment of CVDs are unsatisfactory, despite the advancements in basic research and improvements of clinical therapies [5–8]. This fact, along with the side effects associated with long-term use of synthetic anti-CVD medicines, such as aspirin, statins, and diuretics, implies a tremendous unmet need for exploring complementary and alternative approaches with high safety and efficacy for CVD management [9].

RETRACTED

There is growing interest in naturally occurring products because of their easy availability, low toxicity, and favorable efficiency in reducing the incidence and severity of many health issues [10, 11]. Cinnamon, a popular spice and a type of traditional herbal medicine, has been widely applied to alleviate illness and improve health in Asian countries [12]. Historically, cinnamaldehyde (CA) has been a major active ingredient of the essential oil extracted from the stem bark of cinnamon. In addition to its use as a spice and a flavoring additive in foodstuff and perfumes, CA has been reported to exhibit protective roles against several diseases, including endotoxemia, sepsis, diabetes, ulcerative colitis, and arthritis [13–17]. Accumulating evidence demonstrates that CA can potentially inhibit the initiation and progression of CVDs, and the therapeutic potential of CA is brought by its pleiotropic pharmacological properties involving anti-inflammatory, antiapoptotic, antioxidative, vasodilatory, hypolipidemic, and proangiogenic activities [18–23]. For instance, oral gavage of CA alleviated the progression of plaque lesions via inhibiting the systemic inflammation and regulating blood lipid profiles [22]. Another study reported that the severity of cardiac fibrosis was evidently ameliorated after CA administration in fructose-fed rats [19]. This integrated review summarized and evaluated the current knowledge about the cardiovascular protective actions and relevant molecular mechanisms of CA, with the hope to facilitate future development of discovering new anti-CVD candidates with real-world applications.

## 2. Progress in the Pharmacological Characteristics of CA

### 2.1. Chemical Composition of Cinnamon

The genus Cinnamomum, which belongs to the Lauraceae family, consists of nearly 250 species mostly cultured in the East and South Asia. As a generic term, cinnamon mainly contains two plant species Cinnamomum verum and Cinnamomum cassia Blume. Cinnamon is broadly used as a fragrance additive in daily chemical and dietary supplement industries [13, 14]. Of note, cinnamon has obtained a lot of attention in recent years, due to its stated health benefits [12, 24]. It is documented that the volatile essential oils, the major source of CA, are mainly isolated from the dried stem bark of cinnamon, owing that this segment contains the highest content of oils in the plant, up to 2.5% of bark weight [14, 25]. CA, a yellow and viscous aldehyde liquid constituting nearly 90% of the essential oils, was first purified by Dumas and Péligot via steam distillation and then was synthesized by Chiozza in 1850s [15]. With the development of isolation technique and biosynthetic method, it is convenient to obtain CA and its bioactive derivatives possessing excellent cardiovascular protective properties have been found, including 2-methoxycinnamaldehyde, 2-benzoyloxycinnamaldehyde, 2-hydroxycinnamaldehyde, *α*-bromo-4-chlorocinnamaldehyde, and cinnamic acid [26–30]. The chemical structures of CA and the derivatives are presented in Figure 1.

RETRACTED

### 2.2. Physicochemical and Pharmacokinetic Profiles of CA

Extensive research has been conducted to investigate the physicochemical features of CA. Laboratory data has revealed that CA, which naturally exists in *trans*-CA form, is poorly dissolved in water but possesses superior solubility in organic solvents such as ethyl alcohol, acetic acid, and propylene glycol [15, 31]. Furthermore, CA is volatile and can be easily oxidized to cinnamic acid when exposed to an oxygen-owning environment, which makes it unstable in the bloodstream [32]. With a molecular formula of C_9_H_8_O weighing 132.2, CA (or 3-phenyl-2-propenal) displays a relatively low melting point of -7.5°C and a high boiling point of 248°C, determining its liquid form in the daily application [14, 31]. Considering that the pharmacokinetic parameters of medications are vital for the apprehension of functional mechanisms and the guidance of further clinical practice, several scholars have analyzed the pharmacokinetics of CA through multiple detection techniques [31–39] (Table 1). Based on the results of gas chromatography-mass spectrometry, intravenous administration was a preferable mode of bioavailability for CA when compared to the oral route, as reflected by the low AUC_0-*t*_, short *T*_1/2_ and *T*_max_, and high *C*_max_ in the group that adopted intravenous delivery [35]. Another study explored CA distribution in vivo and discovered that CA was rapidly absorbed and distributed in tissues such as the heart, liver, spleen, lung, kidney, brain, stomach, and intestine, reaching the peak levels in most tissues within 6 h after oral gavage of CA. The spleen was reported to be the major tissue possessing relatively high CA concentration, expect for the digestive tract, implicating the regulatory roles of CA in inflammatory responses and immune functions [40]. In terms of metabolic transformations, the stomach, intestine, and liver are the principal parts required for the biological conversion of CA, which is possibly be related to the low bioavailability of oral administration [40, 41]. With a structure of *α*, *β*-unsaturated aldehyde, CA is more prone to oxidization via enzymatic catalysis, followed by degradation to benzoic acid, and ultimately, getting excreted through urine mainly in the form of hippuric acid [42, 43]. Additionally, concentrations of CA and its metabolites in vivo are difficult to determine after 24 h, which indicates CA's properties of rapid elimination from the body without any long-term accumulation [40].

RETRACTED

### 2.3. Drug Carriers of CA

Although CA has been approved as a generally safe compound by the Food and Drug Administration (FDA) in America and Europe, the low aqueous dissolvability, high volatility, and instability of CA weaken its effectiveness and thereby limit its utilization to some extent [13, 14]. Experimental data has revealed that ≥80% of CA was metabolized when it entered the body [42]. From the perspective of the beneficial pharmacological effects of CA, interests in developing drug encapsulation carriers incorporated with CA are gaining great popularity in enhancing the bioavailability and efficacy of CA. For this purpose, vehicle substrates of the delivery system are incorporated into a matrix to produce small capsules that can protect the active compounds from external factors. This approach elevates the water solubility, stability, and circulatory half-life of the entrapped agents in vivo [44]. Some materials with preferred biodegradability, biocompatibility, and nontoxicity have been used as vectors of CA, which include microemulsion, nanoparticle, polymeric micelle, liposome, nanofiber, and liquid crystal gel [45–65] (Table 2). Zhao et al. suggested that CA encapsulated in submicrometer emulsions exhibited higher plasma concentration, faster tissue distribution, and better antitumor effects in rats when compared to CA alone [32]. Similarly, Dong et al. reported that nanogel packaging of CA enabled the controlled release and oxidation inhibition of drug and oxidation inhibition, which consequently increased CA's bioavailability and more effectively promoted cancer cell apoptosis [53]. With the advancement in molecular biology, a large number of bioactive substances, including dextran, silica, chitosan, cyclodextrin, and hyaluronic acid, have been found to synthesize carriers for improving the therapeutic efficacy of CA [46, 48, 51, 53, 60]. Furthermore, other agents such as suberin, polysorbate 80, and egg yolk lecithin have been reported to be effective in increasing the stability of delivery systems [59, 63]. Recently, some studies indicated that the submicron emulsion loading of CA potently alleviated the development of idiopathic pulmonary fibrosis by inhibiting inflammation and oxidative stress [66]. On the other hand, another study demonstrated that cinnamon essential oil entrapped in emulsions exhibited eminent hypolipidemic, hypoglycemic, and antioxidant effects in diabetic rats [67]. Owing to the impellent effects of inflammation, oxidative injury, and lipid and glucose metabolism disorder on CVD progression, these vehicles might also compliment the roles of CA in the treatment of CVDs; however, these notions remain to be established.

RETRACTED

## 3. Protective Activities of CA in the Management of CVDs

### 3.1. Amelioration of Inflammatory Response

Inflammation is recognized as a necessary physiological process of the host in response to pathogen invasion or tissue damage, which ultimately results in restoration of internal hemostasis. Nonetheless, inappropriate inflammation persistence is an obnoxious pathological phenomenon that might stimulate the production of plentiful inflammatory cytokines and then induce tissue destruction and organ dysfunction, eventually leading to severe disorders [68, 69]. Chronic inflammation acts as the key threat in the pathogenesis of CVDs. It is already known that inflammation involves the reactions of different types of cells, among which the macrophages exert principal accelerative roles. On activation by diverse proinflammatory stimuli, macrophages generate an excess amount of cytokines and enzymes by driving intracellular inflammation-associated signaling transduction and inactivating and degrading I*κ*B, followed by the activation of NF-*κ*B which translocate into the nucleus and transcribes a mass of proinflammatory genes [11, 70, 71]. CA was reported to reduce the contents of iNOS and COX-2 in RAW264.7 macrophages and the concentrations of TNF-*α*, NO, and PGE_2_ in a culture media by suppressing LPS-evoked activation of NF-*κ*B [72, 73]. Schink et al. reported a reduction in the level of IL-8 by LPS-stimulated THP-1 cells after pretreatment with *trans*-CA, and the potential mechanism behind this action was possibly due to the drug-induced restraint of TLR4 oligomerization and the subsequent inflammation signal flow, followed by phosphorylation inhibition of Akt and I*κ*B, which retained NF-*κ*B in the cytoplasm in an inactive form [74, 75]. In addition to prohibiting the translocation of NF-*κ*B into the nucleus, *trans*-CA was demonstrated to exhibit inhibitory roles against the DNA-binding activities of NF-*κ*B under the stimulation of inflammation factors [76]. Via inducing the maturation and the release of IL-1*β*, NLRP3 inflammasome serves as a fundamental inflammation-promoting regulator. There was evidence that CA intervention delayed NLRP3/IL-1*β* signal pathway by blocking the succinate/HIF-1*α* axis in macrophages [17]. Moreover, Kim et al. reported that *trans*-CA could mitigate LPS-provoked activation of ERK1/2, JNK, and p38, accompanied by reduction of contents of iNOS, IL-1*β*, IL-6, and TNF-*α* in RAW264.7 cells [77]. Considering that MAPK cascades involving ERK1/2, JNK, and p38 axis are well-established contributors to the development of inflammation, this agent possibly displays anti-inflammatory effects by weakening the activities of MAPKs signaling molecules (Figure 2(a)). Apart from encumbering the production of proinflammatory elements such as TNF-*α*, IL-6, IL-8, NLRP3, and COX-2, CA had been demonstrated to increase the generation of anti-inflammatory cytokines IL-10 and TGF-*β*, partly owing to the facilitation of macrophage polarization toward M2 phenotype and the suppression of M1-related proteins production, although the precise mechanisms remained elusive [78, 79].

RETRACTED

In the pathological niche, proinflammatory mediators induce vascular endothelial cells (ECs) to elaborate many bioactive substances, such as interleukins, prostaglandins, and adhesion molecules. These inflammatory constituents trigger the disorders of biological properties of ECs, which is termed as endothelial dysfunction, an important predisposing risk event contributing to CVD development [80, 81]. Results from Liu et al. demonstrated that the increment of LPS-evoked mRNA and protein contents of IL-1*β*, IL-6, and TNF-*α* in ECs was reversed by preincubation of CA in a dose- and time-dependent manner. The authors further analyzed the mechanisms and found that the transduction blockade of the TLR4/NF-*κ*B pathway was implicated in anti-inflammatory actions of CA [82]. Moreover, CA had been reported to prevent the rise in the concentration of PGE_2_ in IL-1*β*-insulted ECs by decreasing the activity of COX-2 [83]. Moreover, the upregulation of adhesion molecules on ECs leads to excessive recruitment of circulating leukocytes on the endothelial layer and then facilitates their infiltration across the tunica intima and into the subendothelium, where the leukocytes release excessive inflammation effectors that aggravate the vasculature damage [80]. An experiment performed by Liao et al. claimed that the exposure of ECs to CA led to a time-dependent increment in the I*κ*B protein level, followed by the abrogation of NF-*κ*B activation and the expression of inflammatory genes VCAM-1 and ICAM-1, resulting in the disruption of TNF-*α*-initiated monocytes adhesion to the EC monolayer [84] (Figure 2(b)). Interestingly, another scholar uncovered that CA administration could potently suppress VCAM-1 generation by disrupting NF-*κ*B nuclear translocation in umbilical vein ECs insulted by TNF-*α*, without affecting the production of ICAM-1 and the phosphorylation of NF-*κ*B [85]. The discrepancies observed between these two studies might be explained by the differences in the cell types, dosage, and intervention duration of CA and the participating anti-inflammatory signaling cascades.

RETRACTED

Increasing investigations have placed a focus on the involvement of vascular smooth muscle cells (VSMCs) in the development of vascular inflammatory diseases, as there is proof that activated VSMCs display contributing roles to the vessel disorder through producing vast proinflammatory factors [86]. It was clarified that CA had the capacity of antagonizing ox-LDL-elicited inflammation response in VSMCs, as seen by contents decrement of TNF-*α*, IL-6, MCP-1, and NO, which was attributed to CA-induced inhibition of inflammatory signaling pathways containing JNK, p38, and NF-*κ*B [87].

With respect to the anti-inflammatory functions of CA in vivo, several studies were conducted to explore this trait using different animal models. Using ApoE^−/−^ mice with high fat diet (HFD) for 12 weeks to induce atherosclerotic model, Li et al. showed that supplement with CA for consecutive 8 weeks significantly reduced the size of atheroma plaques in the aorta. Furthermore, they observed that CA treatment caused inflammation alleviation in mice, as indicated by phosphorylation reduction of aortic I*κ*B and NF-*κ*B as well as levels decrement of blood IL-6, MCP-1, TNF-*α*, and NO [22]. It is speculated that the antiatherosclerotic actions of CA could be explained by the inflammation suppression at least in part, by the fact that the inflammatory reaction has been illustrated to present indispensable effects in each stage of plaque lesion development. Accumulating statistics manifest that viral infection-triggered inflammation in myocarditis could collapse homeostasis of myocardial cells and arrangement integrity of myocardial tissues, leading to irreversible cardiac injury. It was revealed that intraperitoneal administration of CA to BALB/c mice infected with coxsackie virus B3 obviously reduced the severity of myocarditis, as indicated by abatement of necrosis, calcification, and fibrosis in the heart tissue, which was associated with the amelioration of myocardial inflammation infiltration resulting from CA-elicited inhibition of TLR4/NF-*κ*B cascade transduction and expressions diminishment of target inflammatory molecules including TNF-*α*, iNOS, IL-1*β*, and IL-6 [29, 88]. These in vitro and in vivo studies suggest that the CA's effectiveness in delaying inflammation mainly derives from its abilities in interrupting proinflammatory gene expression via suppressing upstream NF-*κ*B activation.

RETRACTED

### 3.2. Improvement of Oxidative Stress

Accumulating evidences support that occurrence of oxidative stress is either due to the overproduction of reactive oxygen species (ROS) or impairment of the antioxidant defense system, which leads to an imbalance between oxidants and ROS scavengers tilting toward an oxidative status. These free radicals, including superoxide anion, hydrogen peroxide, and hydroxyl radical, could directly induce lipid peroxidation, protein oxidation, and DNA damage, which, in turn, results in abnormalities in the cellular structure and functions, including loss of membrane integrity, disarrangement of the cytoskeleton, alterations in energy metabolism, and cascade signal flow, as well as the onset of apoptosis-related events, thereby giving rise to the vascular and myocardial injury [11, 89]. It was reported that the protective effects of CA could, to some extent, be interpreted by its repressive actions on oxidative stress, as reflected by content decrement of oxidation damage biomarker malondialdehyde (MDA) in the circulation of HFD-fed mice with plaque regression following CA administration [22]. This observation was confirmed by another independent study implemented by Nour et al., wherein oral gavage of CA to rabbits fed with a high-cholesterol diet for 4 weeks inhibited the development of atherosclerosis. Meanwhile, they showed that CA treatment could effectively lead to a significant decrease in the levels of MDA and myeloperoxidase (MPO) and an increase in the activities of enzymatic antioxidants superoxide dismutase (SOD) and catalase (CAT) in the aortic tissues, respectively [90]. Concerning the regulatory roles in the redox condition of vascular cells, CA could normalize the contents of ROS and MDA in ox-LDL-stimulated ECs by enhancing the level of SOD via activating nuclear factor erythroid-2-related factor 2 (Nrf2), an important transcriptional factor responsible for the expression of antioxidative genes, as reported by Li and colleagues [91]. In agreement, evidence from in vitro experiments attributed antioxidative abilities of CA to its contributing roles in facilitating the transduction of the p38 pathway and the activation of Nrf2, accompanied by generation of antioxidant defense enzyme heme oxygenase (HO-1) in ECs irritated by H_2_O_2_ [85].

RETRACTED

Previous studies have indicated that one essential reason why hyperglycemia is believed to be implicated in the etiology of CVDs is accounted for its inducible capacity in favoring oxidative stress. Advanced glycation end products (AGEs), formed by nonenzymatic reactions of glycolysis intermediates with proteins and/or lipids, are capable of increasing intracellular ROS level by interacting with the receptors (RAGE) which, in turn, activate NADPH oxidase (NOX), the primary enzyme responsible for ROS biosynthesis [92, 93]. Some scholars certified that CA produced inhibitory roles in the transduction of AGEs/RAGE/NOX cascade and sequentially improved the ROS overload in a hyperglycemic environment [94]. Moreover, through elevating the expression of antioxidant substances including HO-1, NADPH dehydrogenase quinone 1 (NQO1), CAT, and glutathione peroxidase 1 (GPX1) via strengthening the activity of the Nrf2 signaling pathway, CA alleviated high glucose-induced oxidative damage on ECs and vascular walls, apart from reducing the activities of NOX p22 and p47, as demonstrated by arterial relaxation and remodeling alleviation [95, 96].

After the treatment through reperfusion strategies like stent angioplasty and intravascular thrombolysis, oxygen and other nutrients in the blood swarm into the myocardium previously supplied by an obstructed artery, which elicits an enormous burst in the ROS activity that exceeds the defensive capacity and then cause an undue formation of ROS that ultimately results in cell death, known as cardiac ischemia/reperfusion (I/R) injury [97, 98]. Results from Sedighi et al. showed that the serum activities of SOD, CAT, and GPX were increased and that the concentrations of MDA and lactate dehydrogenase (LDH) were decreased in the presence of CA, followed by a reduction of the infarct size, cTnI level, and duration of arrhythmias in rats suffering from myocardial I/R damage [99]. Further investigations on the potential mechanisms uncovered that CA might mitigate oxidative stress-induced I/R injury by activating Nrf2/HO-1 and Akt/PPAR*α* axis that were responsible for ROS scavenging and suppressing TLR4/NOX4 cascade participating in ROS generation, respectively, thereby lowering ROS-induced NF-*κ*B activation and expression of downstream cytokines participating in cardiomyocyte impairment [18, 95, 96]. In the animal models of cardiac injury evoked by isoproterenol, LPS, and fructose, the therapeutic actions of CA were focused on improving the oxidative status by restraining the ROS producers NOX and xanthine oxidase (XOD) and increasing the levels of antioxidant enzymes SOD, GSH, and CAT, which, in turn, hampered the signal flow of inflammation-related pathways involving JNK, ERK1/2, p38, and TLR4/6-IRAK4/1 axis, eventually causing expression decline of cytotoxic target effectors, such as TNF-*α*, IL-6, NLRP3, and IL-1*β* [18, 19, 100] (Figure 3). An increasing number of studies document that ROS functions as an agonist of inflammation-associated signaling pathways and that antioxidants are highly efficient in retarding the inflammatory response. Accordingly, CA is likely to interfere with oxidative stress-provoked cardiovascular injury via regulating distal inflammation signaling cascades.

RETRACTED

### 3.3. Regulation of Blood Lipid and Glucose Metabolism

The perspective that atherosclerosis is regarded as a dyslipidemia-related illness has garnered concern because lipid metabolism dysfunction manifests indispensable effects in each stage of plaque lesions and strategies, therefore extenuating dysfunction of lipid metabolism is effective for the treatment of atherosclerosis [80]. It was indicated that CA repressed the increase in the levels of TG, TC, and LDL-C in HFD-induced ApoE^−/−^ mice, accompanied by a reduction of the atherosclerotic lesion size, which might be due to CA-evoked inhibition of lipid deposition and resultant foam cell formation in the subendothelium. This result conformed to those obtained from other studies involving atherosclerotic animal models demonstrating that CA-elicited protective effects were at least partly linked to the actions of improvements in the lipid profiles [22, 90]. Moreover, another mechanism underlying CA-induced delayed generation of foam cells was that CA weakened activation of the ox-LDL-induced NF-*κ*B pathway and downstream expression of LOX-1 required for devouring oxidized lipoproteins [87]. As is already known, hyperlipidemia results from an imbalance between lipid generation and elimination, and AMPK, a serine/threonine protein kinase, serves as an indispensable cellular energy sensor responsible for multiple metabolic processes including lipid anabolism and catabolism [101]. It had been documented that CA administration induced fatty acid oxidation and halted its synthesis in 3T3-L1 adipocytes via activating AMPK, followed by the inhibition of SREBP1c-FAS/SCD-1/GPAT and phosphorylation of ACC [102]. In terms of other relevant bioactive proteins, the increase in the levels of HSL, DGAT2, and PNPLA2 promoting lipolysis and the reduction in the contents of PLIN, FGF21, aP2, and GPD preventing lipolysis were seen in mature adipocytes treated with CA [103, 104]. Moreover, there was evidence uncovering that CA was capable of enhancing the PKA/p38 MAPK pathway activity to facilitate fat consumption and diminishing the PPAR-*γ* and C/EBP*α* expression to reduce fat accumulation in adipocytes [102, 105]. In addition to mediating the metabolic events of adipose cells, CA was found to directly regulate the functions of signal molecules implicated in lipid metabolism in hepatocytes, as reflected by content elevation of phosphorylated AMPK and level decrement of SREBP1c/ACC, whereas the SREBP2 axis, an AMPK target pathway, and its downstream effectors, including HMG-CoA associated with cholesterol production and LDLR implicated in cholesterol ejection, displayed no alteration in the expression levels of CA-fed rat hepatocytes [106]. Considering that the liver acts as the main organ responsible for energy substance metabolism, CA probably exerts cholesterol-lowering roles via affecting the signaling networks in hepatic cells, and elucidating the inner mechanisms is beneficial for paving the way for clinical usage of CA in the management of hypercholesterolemia-triggered CVDs.

RETRACTED

A considerable amount of data exists indicating that hyperglycemia as a critical contributor to the pathogenesis of several CVDs such as atherosclerosis, myocardial infarction, hypertension, and cardiomyopathy. Primarily, by means of favoring inflammation reaction and oxidative stress, high blood glucose causes structural and functional damage to diverse cell types such as vascular ECs, VSMCs, circulating monocytes, and myocardial cells, ultimately leading to disorders of the cardiovascular system [107, 108]. Considering the antihyperglycemic potential of CA as previously reported, the glucose-modulating effects of CA were likely to account for its protective roles against CVDs to some extent. With respect to the hypoglycemic mechanisms, CA was found to boost cellular uptake of glucose and glycogen biosynthesis and improve insulin resistance and dysfunction of pancreatic islets [15, 109]. Specifically, via controlling the upstream signaling cascades including PPARs/RXRs, IRS-1/PI3K/Akt, AMPK, retinol binding protein 4, and PGC-1*α*/MEF2 which were implicated in GLUT4 expression and membrane translocation, the treatment with CA overtly enhanced glucose ingestion and insulin sensitivity in adipose and muscle tissues, thereby leading to the decrement of blood glucose content and HOMA-IR index [94, 110–112]. Considering the excessive gluconeogenesis and insufficient glycogen synthase occurred in the liver of diabetic subjects, CA had been reported to ameliorate glucose metabolism via reversing this disorder through reducing PEPCK and G6Pase activities and strengthening the GYS-2 and PK activities [103, 113] (Figure 4).

RETRACTED

### 3.4. Inhibition of VSMC Proliferation and Migration

Currently, there has been growing attention paid to immoderate proliferation and migration of VSMCs due to their inducible roles in the development of CVDs. Exposed to varying stimuli, VSMCs with a quiescent pattern acquire activated properties which are characterized by undue growth and movement to target regions to exacerbate tissue hypertrophy, extracellular matrix (ECM) degradation, and remodeling, thereby accelerating the occurrence of several CVDs like restenosis after angioplasty, pulmonary arterial hypertension (PAH), and aortic dissection [86, 114]. By reducing the content of proliferating cell nuclear antigen (PCNA) related to the S phase of cell cycle transition, CA suppressed VSMC proliferation triggered by ox-LDL, by the fact that valid progression of cell cycle was fundamental for the proliferative process [87] (Figure 5). With regard to CA-driven antiproliferative mechanisms, Kwon et al. illustrated that cinnamon extracts containing CA and its derivations probably disrupted the activities of mitosis-related signal molecules including PLC*γ*1, AKT, JNK, and p38 MAPK to cause cell cycle arrest at G0/G1 and S phase in growth factor-stimulated VSMCs, as indicated by decreased expressions of cyclin D1/E and CDK2/4 and increased levels of p21 and p27 [115]. It is declared that matrix metalloproteinases (MMPs) belong to a group of endopeptidases cleaving ECM constituents and facilitating VSMC mobilization. The reduced migratory abilities were seen in ox-LDL-elicited VSMCs after intervention with CA, which was attributed to drug-induced MMP-2 level diminution by abating p38, JNK, and NF-*κ*B pathway transduction [87]. Meanwhile, a decrease in MMP-2 content and NF-*κ*B activation within aortic tissues was observed in the atherosclerotic mice upon CA gavage [22]. Another study revealed that CA was beneficial for improving the neointimal hyperplasia after balloon injury in diabetic rodent models by activating Nrf2 axis, accompanied by inhibition of VSMC proliferation and migration, which further confirmed the protective effects of CA against VSMCs-driven disorders [116]. Moreover, monocrotaline was reported to trigger PAH, augment myofibril stiffness, and cause an elevation in right ventricular (RV) pressure overload, while CA was capable of inhibiting the monocrotaline-induced increase in RV systolic pressure via ameliorating the RV fibrosis [117]. However, whether CA attenuated the PAH development to improve RV pressure overload was unknown. Considering that uncontrolled growth and mobilization of VSMCs are highly implicated in the progression of PAH, exploring the regulatory roles of CA in pathological processes of this disease might be of great value for the management of PAH.

RETRACTED

### 3.5. Alleviation of Myocardial Fibrosis

In response to cytokines or ROS-evoked injury, cardiac fibroblasts undergo a programmed conversion into myofibroblasts which release numerous endogenous substances, particularly collagen fibrils, resulting in redundant ECM recruitment and deposition, a process termed myocardial fibrosis. Interest in cardiac fibrosis has increased since the discovery of its contributing properties in deteriorating the reduction of myofiber compliance and exacerbating the dysfunction of heart contraction and dilation [118]. Several studies have ascertained that a variety of biomacromolecule-mediated signals participate in the pathophysiological course of myocardial fibrosis, among which TGF-*β* is a crucial initiator [119]. Kang and collaborators, by Masson trichrome staining, determined that fructose-induced cardiac fibrosis was markedly improved by CA. They further stated that the antifibrotic capacities of CA might be linked to the blockade of the ROS-CD36 axis, followed by TLR4/6-IRAK4/1-NLRP3 cascade retardation and subsequent inactivation of TGF-*β*-mediated Smad2/3 and Smad4 pathways [19]. Moreover, the potential of CA to directly encumber the proliferation and activation of TGF-*β*-induced myocardial fibroblasts was verified by a prominent reduction in the expression of Ki-67 and *α*-SMA. Further amelioration in the level and accumulation of collagen-I/III in the ventricle was observed. The inner mechanistic analysis manifested that calcitonin gene-related peptide- (CGRP-) dependent restraint of the TGF-*β*/NF-*κ*B signaling pathway might account for CA-elicited fibrosis-inhibiting actions [117]. Owing to the involvement of MAPKs in the pathogenesis of myocardial fibrosis and hypertrophy, CA application showed inhibitory effects on cardiomyocyte enlargement, myocardial fibroblasts growth, and collagen secretion, partly by weakening the MEK1/2-ERK1/2 signal pathway [120–122]. During the development of cardiac fibrosis, stromal cells arise from the transdifferentiation of vascular ECs are considered to play contributing roles via favoring profibrotic factors production and ECM accumulation. By the suppression of the TGF-*β*/Smads pathway, the treatment of CA potently increased the contents of CD31 and CD34 and vessel density and decreased the levels of *α*-SMA and vimentin in the heart tissue of mice irritated by pressure overload, suggesting the CA-evoked antagonistic effects on ECs transdifferentiation to stromal cells [123]. It is noteworthy that at the early stage of postmyocardial infarction, moderate cardiac fibrosis is profitable for improving patient prognosis via maintaining structural integrity and compensating for the functional deficiency of the heart. CA had been proved to accelerate myofibroblast formation in cardiac tissues upon MI injury and activation of the Ca2+ influx-CaN-NFAT pathway was likely to be implicated in this fibrotic actions [124]. Thus, it could be inferred that the regulatory roles of CA in myocardial fibrosis vary according to the specific conditions of the diseases, ultimately improving the process of blood pumping, which implies that CA displays a good prospect in the prevention and treatment of cardiac failure.

RETRACTED

### 3.6. Promotion of Vascular Dilation

Temporary vascular contraction is a common physiological reaction seen in strengthening body vigilance and adaptability under stress stimulation. However, persistent vasoconstriction is detrimental to the functioning of internal biological networks, since it induces blood pressure elevation or vasospasm-related tissues ischemia. A series of research findings have identified VSMCs as the chief executors controlling vessel contraction and relaxation. With exposure to both exogenous and endogenous irritants, the myosin and actin in VSMCs undergo conformational changes that modulate the performance of myofilament sliding essential for the process of vasomotion [114, 125]. In vitro, CA was found to induce the relaxant response in vasculatures of different areas including coronary artery, thoracic aorta, and mesenteric artery [21, 93, 126]. This was further verified by in vivo studies suggesting that increased blood pressure evoked by hyperglycemia in rats was recovered via CA intervention [127, 128]. In light of the eminent vasorelaxant actions of CA, several researches were conducted to disclose relevant potential mechanisms, which showed that the activation of Nrf2 and eNOS in ECs played important roles. It was elucidated that excessive ROS triggered the degradation of NO, and the enhanced activity of Nrf2 was capable of mediating the production of antioxidant genes HO-1, NQO1, and CAT and then preventing NO depletion [95]. Since eNOS served as the main NO-producing enzyme, upregulation of Nrf2 and eNOS was profitable for preserving the NO level, thereby favoring this factor diffusion into adjacent VSMCs where NO activated sGC/cGMP/PKG axis associated with phosphorylation of functional proteins promoting vasorelaxation [11, 93, 129]. As for other mechanisms underlying vasodilator properties of CA, blockade of Ca2+ influx and intracellular Ca2+ release and improvement of K+ channels functionality in VSMCs were involved [21, 130, 131] (Figure 6). However, evidence had also suggested that ROS exerted positive roles in facilitating CA-mediated cerebral arterial dilation, as vindicated by transduction suppression of CGRP-PKA and NO-PKG cascade located in the interface between neurons and VSMCs under antioxidant administration [132, 133]. A possible explanation for such a finding might be that CA produced vasorelaxant functions varying according to the surroundings. Furthermore, moderate oxidative stress was beneficial to increase blood supply in the brain tissue for avoiding damage in response to ischemic events. This, together with the recent data that *trans*-CA alleviated cardiac hypertrophy by improving tubulin detyrosination via regulating the SOCE signaling pathway and STIM1/Orai1 translocation, indicated that there were probably unknown mechanisms by which CA elicited epigenetic changes within the contractile proteins to display vasodilator abilities [134].

RETRACTED

### 3.7. Suppression of Platelet Activation and Aggregation

Compelling evidence has highlighted the paramount hazardous characteristics of thromboembolic diseases to human health, due to their close relationship with disability and mortality worldwide. During the process of thrombosis, platelet activation and aggregation are identified as the initiating steps contributing to the development of this pathological disorder, emphasizing antiplatelet medications as the key means for minimizing the risk of these ischemic and anoxic events [135, 136]. In view of the prothrombotic actions of ADP, collagen, arachidonic acid, thrombin, TXA_2_, and TXB_2_, CA was discovered to weaken platelet activation and aggregation induced by the above mentioned cytokines, which was partly attributed to the drug-evoked effects on synthesis inhibition and receptor antagonism of these bioactive substances [137–140]. Moreover, the activation of the eNOS/NO pathway in ECs and the amelioration of phospholipase C/Ca^2+^ influx signaling axis in platelets might be other mechanisms underlying CA's aggregation-abrogating capacities in the bloodstream, owing that the elevation of NO derived from proximal vascular ECs and the decrement of Ca^2+^ content uptake in the platelet triggered the activation of factors like cGMP possessing antiaggregative behaviors and lowered the activity of enzymes including MLCK favoring the onset of aggregation, respectively [93, 95, 141]. Additionally, cinnamic acid treatment was found to abate the generation of TNF-*α*-stimulated tissue factors in ECs through disrupting the NF-*κ*B signal pathway [30]. As cinnamic acid acts as the primary metabolite of CA and the tissue factor is a vital protein implicated in the process of intrinsic hemostasis pathway, there is a possibility that CA plays anti-inflammatory actions to prohibit tissue factor-irritated activation of platelet (Figure 7). From the perspective of thrombolysis in vivo, CA intervention obviously decreased the rate of acute pulmonary thromboembolic death and reduced thrombus weight in the arteriovenous shunt thrombosis model, further demonstrating the safety and efficacy of CA [137, 138].

RETRACTED

### 3.8. Modulation of Cellular Apoptosis

Statistics from laboratory investigations endorse the notion that cellular senescence and programmed apoptosis are crucial for an organism to sustain internal homeostasis; yet, excessive apoptosis of ECs and cardiomyocytes have been intimately related to the pathogenesis of CVDs [80, 81, 142]. In detail, ECs, forming the lining of blood vessels, produce and release diverse active mediators to maintain vasculature tension and integrity, regulate platelet adhesion, balance oxidative stress, and prohibit inflammation response. Cardiomyocytes, acting as the “core engine,” exhibit irreplaceable effects on life activities by pumping blood throughout the body. When these cells are subjected to continuous proapoptotic stimuli, their structure and functions get injured, leading to the development of atherosclerosis, thrombosis, and heart failure [11, 18]. It had been unveiled that CA offered protective roles against EC apoptosis under the environment of oxidative stress and the inner mechanisms were associated with CA-triggered activation of the Nrf2 signaling axis and restraint of NAPDH activity, accompanied by a decline in the intracellular ROS level, restoration of the mitochondrial membrane potential, and alleviation of cytochrome c leakage into the cytosol. These events, in turn, caused transduction blockade of the caspase-related cascade promoting apoptotic cell death [85, 95, 96]. Moreover, given that the ratio of Bax/Bcl-2 participating in the activation of caspase-9/-3 was upregulated by the TLR4/NF-*κ*B pathway and downstream PARP acting as apoptosis executor was decreased by eNOS/NO signaling separately, CA-induced suppression of TLR4/NF-*κ*B and enhancement of eNOS/NO might further confirm its potent prosurvival behaviors against the intrinsic apoptotic pathway in ECs [82, 143]. There was evidence that LPS-evoked cardiac damage was improved by CA treatment, which, to some extent, ascribed to the disruption of proapoptotic signal flow provoked by oxidative stress and inflammatory factors, as seen by activity inhibition of the TLR4/NOX4 and MAPKs/NF-*κ*B pathway in cardiomyocytes [18]. Furthermore, Zheng et al. proved that CA preconditioning protected myocardial cells from ischemia/hypoxia-induced apoptosis via decreasing the expression of Bax and caspase-3 and elevating Bcl-2 level in a PI3K/Akt axis activation-dependent way [20] (Figure 8). It was worth noting that CA conveys motivated functions in favoring apoptosis of tumorous cells through modulating certain molecular pathways such as Wnt/*β*-catenin, PERK/CHOP, and AMPK/mTOR [144–146]. Although past studies on CA-induced double-faced impacts on apoptosis regulation are scarce, it could be supposed that drug dosage and application time, genetic phenotype, redox balance, and signal network mediation are likely to be responsible for CA-related vascular protective and antineoplastic effects. These results, in accordance with the findings that CA was capable of accelerating angiogenesis in noncancerous tissues compensating for ischemic injury while hindering angiogenesis in cancerous tissues aggravating malignant metastasis, indicate that CA has considerable potentials to present as the alternative and adjuvant avenue for improving cardiovascular damage evoked by chemotherapy [23, 146, 147].

RETRACTED

## 4. Other Recent Advances in the Mechanisms of CA against CVDs

With the in-depth understanding of pathogenic courses of CVDs, several molecular actions are newly deemed to be implicated in the regulation of disease development, such as organelle autophagy, endoplasmic reticulum stress, gut microbiota mediation, and ion metabolism [148–151]. Currently, there is a continuing rise in these activities as the promising targets of CA applicable to the cardiovascular system protection upon harmful irritants.

It is revealed that autophagy, featured by a catabolic process degrading intracellular components in a lysosomal dependent manner, is essential for cellular homeostasis and survival [148]. Zhao and colleagues reported that CA repressed hyperactive autophagic actions caused by oxidative stress and inflammation reaction to mitigate organelle overdigestion and maintain cellular integrity, then delaying occurrence of myocardial death stimulated by LPS [18]. Another study showed that obesity-induced autophagy depression in hepatocytes was enhanced by CA gavage, followed by the amplification of hepatic lipid-lowering capacities and the improvement of dyslipidemia in the circulation [106].

When the cells are subjected to adverse threats, numerous unfolded and misfolded proteins assemble in the endoplasmic reticulum (ER) to initiate a series of molecular reactions toward restoring the normal functions of ER, which is defined as ER stress [149]. CA had been reported to alleviate the activation of agonists involved in lipid synthesis by weakening the ER stress in the liver [106]. Additionally, because of the pivotal roles of ER stress in apoptosis progression, the antiapoptotic mechanisms in ECs and cardiomyocytes exerted by CA might be relying on ER stress modulation to some extent, which warrants further investigation [145].

RETRACTED

The immunoreaction acts as the defensive and adaptive conduct for eliminating exogenous and endogenous stimuli in vivo by cooperation of multiple cells and cytokines. Statistics have emerged that exorbitance and misrecognition of the immune system is associated with the development of atherosclerosis and myocarditis [80, 152]. Given that CA possesses immunoregulatory effects including influencing T-cell differentiation and proliferation, regulating monocyte phenotype transformation, and affecting expression of surface antigens, costimulatory molecules, pattern recognition receptors, and complement receptors, figuring out the implication of immunomodulation in CA-elicited cardiovascular protection is worthy [153–156].

As previously portrayed, dysfunction of the gut microbiota is detrimental for the normal operation of physiological processes in vivo, leading to energy metabolism disorder, arterial wall malfunction, myocardial fibrosis, and so on [157]. Results from Zhao et al. indicated that CA intervention reversed level increase of blood glucose in mice under the hyperglycemic condition, through ameliorating imbalance of intestinal flora [158]. It is also plausible that one of the cardioprotective mechanisms of CA might be linked to mitigation of gut microbiota alteration; hence, the forward exploration is needed.

Recently, interest in trace elements has elevated since their abilities to induce a multitude of microcosmic events affecting cell fate, particularly ferroptosis, an iron-dependent mediated form of cell death [151]. Bioinformatic data predicted that CA probably alleviated intracellular iron shortage to inhibit pulmonary vascular remodeling and reduce pulmonary artery pressure, then postponing the deterioration of PAH [159]. As the contribution of ferroptosis regulation to the pharmacological benefits of CA is largely unknown, detailed basic researches are rewarding to be employed for determining whether CA diminishes vascular injury by improving the activation of ferroptosis.

Noncoding (nc) RNAs, comprising microRNAs, long noncoding (lnc) RNAs and circular RNAs, are a group of bioactive factors regulating gene expression at the post-transcriptional level to cause translational enhancement or repression, without clear potentials to encode polypeptides [160]. Administration of CA dramatically restrained inflammatory responses in mice suffering from ulcerative colitis through regulating the expression of miR-21, miR-155, and lncRNA H19 and MIAT, as proved by contents reduction of TNF-*α*, IL-1*β*, IL-6, COX-2, and NLRP3 [16, 161]. It is suggested that above miRNAs and lncRNAs play crucial roles in the inflammation development of cardiovascular tissues, implying that controlling their levels has great possibility to be another target for CA to the management of inflammation-related CVDs [162–165].

RETRACTED

Distributed in multifarious organs including the brain, skin, vasculature, and heart, transient receptor potential ankyrin-1 (TRPA1) is expressed as a six-transmembrane nonselective cation channel with a high calcium permeability and considered to be a signal-carrying messenger activated by physical and chemical products, among which CA serves as an important external agonist [166]. Emerging attention is paid to the signaling network containing TRPA1 because diverse therapeutic effects following CA-triggered TRPA1 activation have been established, such as vasodilation promotion, inflammation restraint, apoptosis abolishment, and immune regulation [79, 133, 143, 154]. It remains obscure whether CA interferes with diseases development predominately or solely depending on mediating TRPA1 activity, illuminating this confusion would provide a feasible direction for thoroughly recognizing the cardiovascular protective mechanisms of CA and lay the theoretical foundation for the compound applied in CVDs prophylaxis and treatment.

## 5. Potential Risks of CA

However, the current knowledge on the safety, stability, and bioavailability of CA is limited. Although herb medications have been widely applied in disease treatment for a long time, the appearance of side effects such as hepatic and renal damage are not rare. Thus, investigating whether CA exhibits excellent safety in clinical application is of high priority. According to the FDA of multiple countries, CA is proved as no safety concerns at doses of not exceeding daily acceptable consumption, whereas higher and nonnutritional intake of CA is prone to the appearance of genetic alteration and hepatotoxicity [15]. It is deciphered that CA administration in cellular and animal studies conducted at a specific period of time determines its absence of toxicity and carcinogenicity, the possible effects of this compound regarding long-term duration and other delivery routes are still vague [167, 168]. The results of previous animal studies indicate that CA has a wide spectrum of efficacious dosage against CVDs, ranging from 5 mg/kg to 200 mg/kg. In terms of the upper tolerant level, CA is reported to possess an oral lethal dose scope from a low of 600 mg/kg body weight to a high of 3400 mg/kg body weight in diverse individuals. For instance, the occurrence of hepatotoxicity of CA uptake dosage in rats and mice is 1100 mg/kg/body weight and 850 mg/kg/body weight, respectively [15]. Moreover, it has been reported that CA has a high volatility, indicating the instability of this drug during the process of isolation and delivery. Considering the hydrophobic property of CA, exposure of this agent to aqueous solutions usually lead to a poor bioavailability (approximately 20%). Despite that CA easily dissolve in organic solvents, the toxicity of which is a major concern. It has been demonstrated that several biomaterials including liposomes, nanoparticles, and hydrogels possess favorable biocompatibility, biodegradability, and low immunogenicity properties and are found to encapsulate drugs to act as delivery carriers. By loading in biomaterials, the bioactive compounds could overcome own shortcomings including poor water solubility, low retention, burst release, and rapid clearance, accompanied by acquisition of desirable stability and bioavailability [44]. There is evidence that CA encapsulated in certain nanocarriers obtains decreased cytotoxicity and increased bioavailability, yet whether these constituents possess sanative roles in inhibiting CVDs development is outside the scope of existing investigations [31, 32]. As such, further in vivo experiments should be undertaken for purpose of optimizing the pharmacodynamics and pharmacokinetics associated with curative potentials of CA. In addition, growing clinical trials are advocated to offer scientific basis for the safe and effective use of CA in the management of CVDs.

RETRACTED

## 6. Conclusion

Multiple lines of evidence support that CVDs, with complicated etiology and upward trend in the incidence year by year, are a cluster of pathological factors that impair the power source and mobile carrier of blood flow and seriously harm the physical and mental health of mankind [1, 2]. A nonnegligible reason for this situation is the limitation of therapy and the undesirable adverse effects of drugs used in the clinical practice. Nowadays, much emphasis has been placed on herbal products and dietary ingredients due to the valuable effects of constituents derived from them on disease management. CA, commonly used as a flavoring and fragrance agent, is a naturally occurring phytochemical and has been documented to possess wide spectrum of anti-CVD properties over the past decades [9, 11, 15]. In this review, we summarize and evaluate CA-elicited therapeutic roles against cardiovascular disorders via diverse pharmacological activities, among which inhibition of inflammation and oxidative stress, improvement of lipid and glucose metabolism, regulation of cell proliferation and apoptosis, suppression of cardiac fibrosis, and platelet aggregation and promotion of vasodilation and angiogenesis are involved (Figure 9). Moreover, a phenomenon that a few molecular actions induced by CA lead to dissimilar outcomes between two types of disease models is discussed, differences in cell type and phenotype, compound dosage and duration, and signaling transduction regulation might be the plausible interpretation, which deserve intensive laboratory probe. Meanwhile, in-depth analyses so far have demonstrated that CA is likely to produce cardiovascular benefits through several equivocal mechanisms including mediating autophagy and ER stress, improving gut microbiota and immune homeostasis and affecting ion metabolism, ncRNA expression, and TRPA1 activation, ascertaining their reliability is of vital importance for providing novel insights into the protective effects exerted by CA on alleviating the CVD development.

RETRACTED

## Figures and Tables

**Figure 1:** The chemical structures of CA and its derivatives.

**Figure 2:** (a) The potential signal cascades regulated by CA for affecting inflammation development in macrophages. CA inhibits the expression of proinflammatory factors via suppressing the activities of NF-*κ*B and HIF-1*α* and facilitates M2 phenotype transformation via regulating EZH2 activity. LPS: lipopolysaccharide; TLR4: Toll-like receptor 4; MyD88: myeloid differentiation primary response 88; TRIF: Toll/IL-1R domain-containing adaptor-inducing IFN-*β*; TAK1: TGF-*β*-activated kinase 1; TBK1: tank binding kinase 1; NF-*κ*B: nuclear factor of *κ*B; IRF3: interferon regulatory factor 3; GPR91: G-protein-coupled receptor 91; EZH2: enhancer of zeste homolog 2; TRPA1: transient receptor potential ankyrin-1; HIF-1*α*: hypoxia-inducible factor-1*α*; H3K27me3: histone H3 lysine 27 trimethylation; ARG-1: arginase-1; NLRP3: NOD-like receptor family pyrin domain containing 3; IL-1*β*: interleukin-1*β*; TGF-*β*: transforming growth factor-*β*; JNK: c-Jun N-terminal kinase; ERK1/2: extracellular signal-regulated kinase 1/2; Akt: protein kinase B; iNOS: inducible nitric oxide synthase; COX-2: cyclooxygenase-2; TNF-*α*: tumor necrosis factor *α*; IFN*β*: interferon *β*. (b) CA exerts beneficial roles against inflammation response in ECs induced by cytokines. NF-*κ*B is regarded as the main target involved in the anti-inflammatory effects of CA. HO-1: heme oxygenase-1; VCAM-1: vascular cell adhesion molecule-1; ICAM-1: intercellular adhesion molecule-1; Nrf2: nuclear factor erythroid-2-related factor 2; AA: arachidonic acid; PGE2: prostaglandin E2.

**Figure 3:** The schematic description of signaling pathways responsible for the actions of CA to alleviate oxidative stress. Activation of multiple membrane receptors increase the activity of NOX which is the main producer of intracellular ROS. Excessive ROS triggers cellular damage by accelerating lipid peroxidation and enhancing signals transduction of inflammatory pathways. CA is capable of improving the imbalance of redox through decreasing the activities of NOX and XOD and increasing the activation of Nrf2 axis. PUFA: polyunsaturated fatty acids; MCI: mitochondrial respiratory chain complex I; TXNIP: thioredoxin-interacting protein; AGEs: advanced glycation end products; RAGE: receptor of AGEs; ox-LDL: oxidized low-density lipoprotein; LOX-1: lectin-like oxidized low-density lipoprotein receptor-1; NOX: NADPH oxidase; XOD: xanthine oxidase; IRAK1: interleukin receptor-associated kinase 1; ROS: reactive oxygen species; MDA: malondialdehyde; PPAR*α*: peroxisome proliferator-activated receptor-*α*; BTK: Bruton's tyrosine kinase; Keap1: Kelch-like ECH-associated protein 1; RXR: retinoid X receptor; MPO: myeloperoxidase; CAT: catalase; SOD: superoxide dismutase; NQO1: NADPH dehydrogenase quinone 1; GPX1: glutathione peroxidase 1; *γ*-GCS: *γ*-glutamyl cysteine synthetase.

RETRACTED

**Figure 4:** CA reduces the concentrations of circulating lipid and glucose by promoting energy catabolism and weakening its anabolism. SREBP1c: sterol regulatory element-binding protein 1c; FAS: fatty acid synthase; SCD-1: stearoyl-CoA desaturase-1; GPAT: glycerol phosphate acyltransferase; ACC: acetyl-CoA carboxylase; PKA: protein kinase A; C/EBP*α*: CCAAT enhancer-binding protein *α*; PLIN: perilipin; FGF21: fibroblast growth factor-21; GPD: glyceraldehyde-3-phosphate dehydrogenase; PPAR*γ*: peroxisome proliferator-activated receptor *γ*; HSL: hormone-sensitive lipase; DGAT2: diacylglycerol O-acyltransferase 2; PNPLA2: patatin-like phospholipase domain containing 2; AMPK: AMP-activated protein kinase; SIRT: sirtuin; PI3K: phosphatidylinositol-4,5-bisphosphate 3-kinase; IRS-1: insulin receptor substrate-1; PGC-1*α*: peroxisome proliferator-activated receptor-gamma coactivator-1*α*; GLUT4: glucose transporter 4; MEF2: myocyte enhancer factor 2; G6Pase: glucose-6-phosphatase; PK: pyruvate kinase; PEPCK: phosphoenolpyruvate carboxykinase; GYS-2: glycogen synthase 2.

**Figure 5:** The possible targets mediated by CA to suppress VSMC proliferation and migration. PDGF-PDGFR signaling and oxidative stress induce activation of downstream pathways associated with the expression of cell cycle proteins, CDKs, and MMPs. The protective mechanisms of CA are attributed to the blockade of PDGFR activation and decrease of ROS level. PDGF: platelet-derived growth factor; PDGFR: PDGF receptor; NOX: NADPH oxidase; LOX-1: LOX-1: lectin-like oxidized low-density lipoprotein receptor-1; PLC*γ*: phospholipase C *γ*; PKC: protein kinase C; MMP: metalloproteinase; MCP-1: monocyte chemoattractant protein-1; Akt: protein kinase B; PI3K: phosphatidylinositol-4,5-bisphosphate 3-kinase; PIP3: phosphatidylinositol (3,4,5)-triphosphate; JNK: c-Jun N-terminal kinase; Keap1: Kelch-like ECH-associated protein 1; Nrf2: nuclear factor erythroid-2-related factor 2; PNCA: proliferating cell nuclear antigen; Rb: retinoblastoma tumor suppressor protein; CDK: cyclin-dependent kinase; Prx1: peroxiredoxin; GCLC: glutamate-cysteine ligase catalytic subunit; SOD: superoxide dismutase; HO-1: heme oxygenase-1.

RETRACTED

**Figure 6:** CA modulates the transfer of messenger molecules to decrease Ca2+ content in VSMCs and then induce the occurrence of vascular dilation. NO and CGRP derived from ECs and neurons enter into adjacent VSMCs for opening specific potassium channel which facilitates outflow of potassium and thus causing the hyperpolarization of membrane, which inhibit the open of voltage gated calcium channel and the influx of calcium. The activation of Ca2+-ATPase and inactivation of IP3R in SR is capable of accelerating Ca2+ in the cytoplasm entry into the SR. CGRP: calcitonin gene-related peptide; SR: sarcoplasmic reticulum; MLCK: myosin light-chain kinase; MLCP: myosin light-chain phosphatase; Akt: protein kinase B; Nrf2: nuclear factor erythroid-2-related factor 2; ROS: reactive oxygen species; eNOS: endothelial nitric oxide synthase; NO: nitric oxide; TRPA1: transient receptor potential ankyrin-1; AGEs: advanced glycation end products; RAGE: receptor of AGEs; NOX: NADPH oxidase; GPCR: G protein-coupled receptor; PLC: phospholipase C; IP3: inositol triphosphate; IP3R: IP3 receptor; PKA: protein kinase A; cAMP: cyclic adenosine monophosphate; AC: adenylyl cyclase; PKG: protein kinase G; cGMP: cyclic guanosine monophosphate; sGC: soluble guanylate cyclase.

**Figure 7:** The regulatory effects of CA on the suppression of platelet activation and aggregation. NO synthesized by eNOS of vascular endothelium diffuses into circulating platelet and further induces the production of cGMP which prohibits the aggregative ability. PLC activation triggers level increase of intracellular calcium and then elevates the activity of MLCK responsible for the activation and aggregation of platelets. IC: inflammatory cytokines; TF: tissue factor; eNOS: endothelial nitric oxide synthase; NO: nitric oxide; cGMP: cyclic guanosine monophosphate; PLC: phospholipase C; MLCK: myosin light-chain kinase; NF-*κ*B: nuclear factor of *κ*B; AA: arachidonic acid; ADP: adenosine diphosphate; TXA2: thromboxane A2; TXB2: thromboxane A2.

RETRACTED

**Figure 8:** CA displays inhibitory roles in cellular death via suppressing the mitochondrial-dependent apoptotic pathway. Oxidative stress and inflammatory cascades induce activities increase of p53 and NF-*κ*B, both of which contribute to level elevation of Bax. While PI3K/Akt and Nrf2 signaling axis induce content increase of Bcl-2 and level reduction of Bax on the membrane, which weaken Cyt C release into the cytosol and then disrupt the activation of caspase-9 and caspase-3. PI3K: phosphatidylinositol-4,5-bisphosphate 3-kinase; Akt: protein kinase B; NOX: NADPH oxidase; Nrf2: nuclear factor erythroid-2-related factor 2; HO-1: heme oxygenase-1; CAT: catalase; GPX1: glutathione peroxidase 1; TLR4: Toll-like receptor 4; JNK: c-Jun N-terminal kinase; ERK1/2: extracellular signal-regulated kinase 1/2; NQO1: NADPH dehydrogenase quinone 1; NF-*κ*B: nuclear factor of *κ*B; eNOS: endothelial nitric oxide synthase; NO: nitric oxide; Bcl-2: B-cell lymphoma 2; PARP: poly (ADP-ribose) polymerase; Cyt C: cytochrome C; Apaf-1: apoptosis protease activating factor-1.

**Figure 9:** The schematic diagram of CA against the pathogenic factors involved in the development of CVDs.

**Table 1:** The in vivo pharmacokinetic features of CA.

Formulation	Sample	Dosage of contained CA	Delivery route	Detection method	Parameters					Ref.
					*T*_max_	*C*_max_	AUC0-t	*T*_1/2_	MRT	
CA	Male F344 rat plasma	250 mg/kg	Oral	HPLC	0.4 ± 0.1 h	1.3 ± 0.2 *μ*g/mL	10.5 ± 1.2 *μ*g·h/mL	—	—	
		500 mg/kg			4.1 ± 0.9 h	2.4 ± 0.4 *μ*g/mL	35.2 ± 1.4 *μ*g·h/mL	11.0 ± 0.6 h	—	[33]
ME-CA		250 mg/kg			1.9 ± 0.5 h	1.2 ± 0.1 *μ*g/mL	14.7 ± 2.0 *μ*g·h/mL	—	—	
		500 mg/kg			2.7 ± 0.8 h	1.8 ± 0.1 *μ*g/mL	36.2 ± 4.2 *μ*g·h/mL	12.0 ± 1.2 h	—	

CA	Male SD rat plasma	20 mg/kg	Intravenous	GC-MS	0.04 ± 0.02 h	547 ± 142 ng/mL	375 ± 83.5 ng·h/L	3.26 ± 2.82 h	0.96 ± 0.21 h	[32]
SME-CA		20 mg/kg			0.04 ± 0.02 h	1052 ± 184 ng/mL	589 ± 59.2 ng·h/L	2.17 ± 0.96 h	0.84 ± 0.14 h	

Guizhi-gancao decoction	Male rat plasma	47 mg/kg	Oral	UPLC-MS/MS	0.2 ± 0.1 h	1.1 ± 0.5 ng/mL	2.1 ± 0.2 ng·h/mL	1.5 ± 0.3 h	—	[34]

CA	Male SD rat plasma	50 mg/kg	Oral	HPLC	0.33 ± 0.05 h	301.6 ± 67.9 mg/L	447.1 ± 3.8 mg·h/L	—	—	[31]
CA-SME		50 mg/kg			1.00 ± 0.13 h	1063.4 ± 165.4 mg/L	1802.2 ± 80.8 mg·h/L	—	—	

CA	Male SD rat plasma	125 mg/kg	Oral	GC-MS	1.8 ± 0.4 h	82 ± 15 ng/mL	677 ± 127 ng·h/mL	6.8 ± 2.6 h	5.8 ± 1.3 h	
		250 mg/kg			2 ± 0.7 h	121 ± 14 ng/mL	1141 ± 265 ng·h/mL	6.2 ± 1.5 h	7.1 ± 1.6 h	[35]
		500 mg/kg			1.6 ± 0.5 h	249 ± 36 ng/mL	1984 ± 531 ng·h/mL	6.7 ± 1.5 h	7.6 ± 0.6 h	
		20 mg/kg	Intravenous		0.03 h	547 ± 142 ng/mL	355 ± 53 ng·h/mL	1.70 ± 0.32 h	0.8 ± 0.2 h	

TCA gel	Male Wistar rat plasma	100 mg/kg	Percutaneous	UPLC	1.83 ± 1.07 h	9.71 ± 5.92 *μ*g/mL	58.4 ± 25.4 mg·h/mL	—	4.52 ± 1.05 h	
TCA V2 phase		100 mg/kg			7.33 ± 3.59 h	8.09 ± 2.16 *μ*g/mL	42.9 ± 29.6 mg·h/mL	—	10.7 ± 2.9 h	[36]
TCA H2 phase		100 mg/kg			1.20 ± 0.46 h	11.33 ± 1.90 *μ*g/mL	94.1 ± 10.9 mg·h/mL	—	6.34 ± 1.34 h	

CA	Male SD rat plasma	250 mg/kg	Oral	HPLC	0.31 ± 0.07 h	70.40 ± 23.91 *μ*g/mL	—	—	2.9 ± 0.71 h	[37]
CA-SEDDS		250 mg/kg			0.92 ± 0.20 h	182.0 ± 29.2 *μ*g/mL	—	—	1.76 ± 0.20 h	

CRO	Male rat plasma	12.52 mg/kg	Oral	UHPLC-MS/MS	1.0 ± 0.0 h	22.7 ± 3.2 ng/mL	131 ± 6.7 ng·h/mL	8.7 ± 0.7 h	—	[38]

SBP	Male SD rat plasma	15.73 mg/kg	Oral	HS-SPDE-GC-MS/MS	0.50 ± 0.23 h	18.76 ± 2.11 ng/mL	262.2 ± 63.9 ng·h/mL	13.3 ± 5.8 h	9.80 ± 0.66 h	[39]

ME-CA: microencapsulated CA; SME-CA: submicrometer emulsion of CA; Guizhi-gancao decoction: a formula consisting of *Ramulus cinnamomi* and *Radix glycyrrhizae*; CA-SME: CA submicron emulsion; TCA: *trans*-CA; TCA V2 phase: a compound contains phytantriol, water, and *trans*-CA; TCA H2 phase: a compound contains phytantriol, triglyceride, water, and *trans*-CA; CA-SEDDS: CA with self-emulsifying drug delivery systems; CRO: *Cinnamoni Ramulus*; SBP: Shexiang Baoxin Pill; *T*_max_: the time to reach *C*_max_; *C*_max_: the maximum plasma concentration; AUC_0-*t*_: area under the curve to termination time; *T*_1/2_: half-life; MRT: mean residence time; HPLC: high-performance liquid chromatography; GC-MS: gas chromatography-mass spectrometry; UPLC-MS/MS: ultraperformance liquid chromatography-tandem mass spectrometry; UPLC: ultraperformance liquid chromatography; UHPLC-MS/MS: ultrahigh-performance liquid chromatography-tandem mass spectrometry; HS-SPME-GC-MS: headspace solid-phase microextraction coupled to gas chromatography-mass spectrometry.

RETRACTED

**Table 2:** The parameters of drug delivery vehicles loading CA.

Formulation	Carrier	Average diameter	Polymer dispersion index	Zeta potential	Entrapment efficiency	Application	Ref.
Nanoparticle	P-SS-D	125 nm	0.16	—	—	Antitumor	[45]
Nanoparticle	Dextran, 10-hydroxy camptothecin	182.3 nm	0.225	-3.86 mV	57.6%	Antitumor	[46]
Nanoparticle	PLGA	130.4 nm	0.512	-3.54 ~ -3.86 mV	—	Antifungal	[47]
Inclusion complex	*β*-Cyclodextrin	2-4 *μ*m	—	—	45.39%	Antioxidant	[48]
Liposome	DSPE-PEG2000-PMB	150~200 nm	0.1 ~ 0.2	0 ~ 10 mV	31.93 ± 0.6%	Antibacteria	[49]
Liposome	Egg yolk lecithin, tween 80, chitosan	550~650 nm	—	60~80 mV	50~60%	Antibacteria	[50]
Nanocapsule	Chitosan	165 ± 6 nm	0.18	42 ± 5 mV	78 ± 3%	Antibacteria	[51]
Nanoparticle	Chitosan	254.66 nm	0.28	15.26 mV	77.3%	Antitumor	[52]
Nanoparticle	MSN@GO-HA	115.59 ± 13.98 nm	0.25 ± 0.02	−27.53 ± 4.56 mV	84.36 ± 3.52%	Antitumor	[53]
Submicrometer emulsion	Soybean oil, egg lecithin, glyceriunm	130 ± 5.92 nm	—	−25.7 ± 6.0 mV	99.5 ± 0.25%	Antitumor	[32]
Nanovesicle	Hyaluronic acid, ethanol	250~350 nm	—	-25 ~ -30 mV	75~ 85%	Antiulcerative colitis	[54]
Liposome	DODAB:MO	545 ± 17 nm	0.46 ± 0.06	48.2 ± 2.1 mV	44.1 ± 2.7%	Antifungal	[55]
Nanoparticle	GNP	326 ± 48 nm	—	−45 ± 1 mV	—	Antibacteria	[56]
Microsphere	PHBV/MBGN	7.2 ± 1.5 *μ*m	0.4 ± 0.1	−21.3 ± 0.5 mV	99.96 ± 0.01%	Antiosteomyelitis	[57]
Nanoparticle	PSCI	123.4 nm	—	-11.4 mV	41.4%	Antitumor	[58]
Liposome	Egg yolk lecithin, tween 80, ethanol	75~ 92 nm	<0.3	—	30~ 40%	Antibacteria	[59]
Nanosphere	SiO_2_, hydrogel	200~ 250 nm	—	5 ~ 15 mV	—	Antiwound infection	[60]
Nanogel	PssNCT	200 nm	0.155 ± 0.016	-25~ 0 mV	86.3%	Antitumor	[61]
Nanoparticle	Hyaluronic acid, mesoporous silica	100 nm	—	12.3 mV	—	Antibacteria	[62]
Nanoparticle	Suberin	80~ 110 nm	0.16~ 0.23	-30 mV	—	Antibacteria, antitumor	[63]
Nanocapsule	LNC	99 ± 6 nm	0.120 ± 0.024	−17.7 ± 2.12 mV	—	Antibacteria	[64]
Nanoparticle	Hyaluronic acid	166.0 ± 9.5 nm	0.198 ± 0.005	—	—	Antitumor	[65]

P-SS-D: an amphiphilic polymer skeletal containing 1,3-dimercapto-2-propanol, 1,3-dimercaptopropane, N,N′-carbonyldiimidazole, DOPA, triethylamine; PLGA: DL-lactide-co-glycolide; DSPE-PEG2000-PMB: a liposomal system containing N-hydroxy succinimide, polymyxin B, 1-(3-dimethylaminopropyl)-3-ethylcarbodiimide, DSPE-PEG2000-COOH; MSN@GO-HA: graphene oxide wrapped mesoporous silica nanoparticles modified with hyaluronic acid; DODAB:MO: a system of dioctadecyldimethylammonium bromide and monoolein; GNP: gold nanoparticles; PHBV/MBGN: polyhydroxybutyrate-co-hydroxyvalerate with mesoporous bioactive glass nanoparticles; PSCI: platelet membrane-coated mesoporous silica nanoparticles; PssNCT: N-isopropylacrylamide-co-CA-co-D-*α*-tocopheryl polyethylene glycol 1000 succinate; LNC: a lipid nanocapsule containing polyxyl 15 hydroxystearate, hydrogenated lecithin, triglycerides.

## Abbreviations

CVDs: Cardiovascular diseases
CA: Cinnamaldehyde
FDA: Food and Drug Administration
NF-*κ*B: Nuclear factor-kappa B
iNOS: Inducible nitric oxide synthase
COX-2: Cyclooxygenase-2
TNF-*α*: Tumor necrosis factor *α*
NO: Nitric oxide
PGE_2_: Prostaglandin E2
LPS: Lipopolysaccharide
IL-8: Interleukin-8
TLR4: Toll-like receptor 4
Akt: Protein kinase B
PI3K: Phosphatidylinositol-4,5-bisphosphate 3-kinase
IL-1*β*: Interleukin-1*β*
NLRP3: NOD-like receptor family pyrin domain containing 3
HIF-1*α*: Hypoxia-inducible factor-1*α*
ERK1/2: Extracellular signal-regulated kinase 1/2
JNK: c-Jun N-terminal kinase
IL-6: Interleukin-6
MAPKs: Mitogen-activated protein kinases
IL-10: Interleukin-10
TGF-*β*: Transforming growth factor-*β*
ECs: Endothelial cells
VCAM-1: Vascular cell adhesion molecule-1
ICAM-1: Intercellular adhesion molecule-1
VSMCs: Vascular smooth muscle cells
ox-LDL: Oxidized low-density lipoprotein
MCP-1: Monocyte chemoattractant protein-1
ApoE: Apolipoprotein E
HFD: High-fat diet
ROS: Reactive oxygen species
MDA: Malondialdehyde
MPO: Myeloperoxidase
SOD: Superoxide dismutase
CAT: Catalase
Nrf2: Nuclear factor erythroid-2-related factor 2
HO-1: Heme oxygenase-1
H2O2: Hydrogen peroxide
AGEs: Advanced glycation end products
NOX: NADPH oxidase
NQO1: NADPH dehydrogenase quinone 1
GPX1: Glutathione peroxidase 1
I/R: Ischemia/reperfusion
LDH: Lactate dehydrogenase
cTnI: Cardiac troponin I
PPAR*α*: Peroxisome proliferator-activated receptor-*α*
XOD: Xanthine oxidase
IRAK: Interleukin-1 receptor-associated kinase
TG: Triglyceride
TC: Total cholesterol
LDL-C: Low-density lipoprotein cholesterol
LOX-1: Lectin-like oxidized low-density lipoprotein receptor-1
AMPK: AMP-activated protein kinase
SREBP: Sterol regulatory element-binding protein
FAS: Fatty acid synthase
SCD-1: Stearoyl-CoA desaturase-1
GPAT: Glycerol phosphate acyltransferase
ACC: Acetyl-CoA carboxylase
PKA: Protein kinase A
C/EBP*α*: CCAAT enhancer-binding protein *α*
LDLR: Low-density lipoprotein receptor
IRS-1: Insulin receptor substrate-1
PGC-1*α*: Peroxisome proliferator-activated receptor-gamma coactivator-1*α*
GLUT4: Glucose transporter 4
ECM: Extracellular matrix
PAH: Pulmonary arterial hypertension
PCNA: Proliferating cell nuclear antigen
PLC*γ*1: Phospholipase C *γ*1
CDK: Cyclin-dependent kinase
MMPs: Metalloproteinases
CGRP: Calcitonin gene-related peptide
eNOS: Endothelial nitric oxide synthase
sGC: Soluble guanylate cyclase
PKG: Protein kinase G
TXA_2_: Thromboxane A2
MLCK: Myosin light chain kinase
PARP: Poly(ADP-ribose) polymerase
ER: Endoplasmic reticulum
TRPA1: Transient receptor potential ankyrin-1.
